RETRACTED

# Tyrosine Nitration of PA700 Links Proteasome Activation to Endothelial Dysfunction in Mouse Models with Cardiovascular Risk Factors

**DOI:** 10.1371/journal.pone.0029649

**Published:** 2012-01-17

**Authors:** Jian Xu, Shuangxi Wang, Miao Zhang, Qilong Wang, Sima Asfa, Ming-Hui Zou

**Affiliations:** 1 Division of Endocrinology and Diabetes, Department of Medicine, University of Oklahoma Health Sciences Center, Oklahoma City, Oklahoma, United States of America; 2 Division of Molecular Medicine, Department of Medicine, University of Oklahoma Health Sciences Center, Oklahoma City, Oklahoma, United States of America; 3 Division of Gastroenterology, Department of Medicine, University of Oklahoma Health Sciences Center, Oklahoma City, Oklahoma, United States of America; University of Hong Kong, China

## Abstract

Oxidative stress is believed to cause endothelial dysfunction, an early event and a hallmark in cardiovascular diseases (CVD) including hypertension, diabetes, and dyslipidemia. However, the targets for oxidative stress-mediated endothelial dysfunction in CVD have not been completely elucidated. Here we report that 26S proteasome activation by peroxynitrite (ONOO^−^) is a common pathway for endothelial dysfunction in mouse models of diabetes, hypertension, and dyslipidemia. Endothelial function, assayed by acetylcholine-induced vasorelaxation, was impaired in parallel with significantly increased 26S proteasome activity in aortic homogenates from streptozotocin (STZ)-induced type I diabetic mice, angiotensin-infused hypertensive mice, and high fat-diets -fed LDL receptor knockout (LDLr^−/−^) mice. The elevated 26S proteasome activities were accompanied by ONOO^−^-mediated PA700/S10B nitration and increased 26S proteasome assembly and caused accelerated degradation of molecules (such as GTPCH I and thioredoxin) essential to endothelial homeostasis. Pharmacological (administration of MG132) or genetic inhibition (siRNA knockdown of PA700/S10B) of the 26S proteasome blocked the degradation of the vascular protective molecules and ablated endothelial dysfunction induced by diabetes, hypertension, and western diet feeding. Taken together, these results suggest that 26S proteasome activation by ONOO^−^-induced PA700/S10B tyrosine nitration is a common route for endothelial dysfunction seen in mouse models of hypertension, diabetes, and dyslipidemia.

## Introduction

Peroxynitrite (ONOO^−^) is formed by the reaction of superoxide anions with nitric oxide (NO) at diffusion-controlled rate. It represents a crucial pathogenic mechanism in CVD when excessively produced [1], [2]. Among many chemical reactions, ONOO^−^ is well known by its impact on proteins through tyrosine nitration and leaving its footprint as 3-nitrotyrosine [2]. Many studies have elegantly demonstrated endogenous ONOO^−^ generation and its diverse downstream targets, such as lipids, DNA, and proteins [2], in CVD. Although the roles of ONOO^−^ in the pathogenesis of endothelial dysfunction and atherosclerosis have been well established, the protein targets of ONOO^−^ in CVD have been largely unidentified.

RETRACTED

The ubiquitin proteasome system (UPS) functions as the major non-lysosomal intracellular proteolytic system responsible for degradation of most proteins, particularly those of short-lived and regulatory nature [3]. The essential role of this system includes control of protein quality, cell cycle, transcription factor regulation, gene expression, cell differentiation, and immune response [4]. Degradation of proteins by the UPS occurs in two steps, including targeting of proteins and successive degradation by the 26S proteasome, the major proteolysis complex in the system. The 26S proteasome is a multi-catalytic protease consisting of a 20S catalytic core and two 19S regulatory particles (PA700) [4]. PA700 is first characterized as an ATP-dependent 20S proteasome activator for 26S proteasome activation [5]. Later, sub-complexes of PA700 important for substrate selection and processing have also been identified [6], [7]. Regardless modes of action, increasing evidence demonstrate that PA700 is crucial in functional regulation of the UPS [8]. Alterations in UPS have been shown to contribute to the pathogenesis of cancer, neurodegenerative, and immune diseases [9]. An emerging role has been implicated in the pathogenesis of atherosclerosis [10].

Endothelial dysfunction, defined by impaired endothelium-dependent relaxation, is an early marker for atherosclerosis. Many of the risk factors such as diabetes, hypertension, and dyslipidemia that predispose to atherosclerosis can also cause endothelial dysfunction, and the presence of multiple risk factors has been found to predict endothelial dysfunction. Available data suggest that oxidant stress-activated 26S proteasome mediated endothelial dysfunction in streptozotocin-induced diabetic mice [11] and angiotensin II (Ang II) induced hypertensive mice [12], as well as in experimental hypercholesterolemia pig [13]. It remained to be established if oxidative stress-activated 26S proteasomes is an early and a common pathogenic phenomenon for cardiovascular risk factors and cardiovascular diseases (CVD). Here we report that ONOO^−^ tyrosine nitrates PA700/S10B resulting in activation of 26S proteasome and consequent endothelial dysfunction in mouse models of diabetes, hypertension and dyslipidemia.

RETRACTED

## Materials and Methods

### Materials

Mouse GTPCH I antibody was purchased from Ascenion GmBH (Munich, Germany); ubiquitin antibody from Santa Cruz Biotechnology (Santa Cruz, CA); mouse PA700/S10B antibody from Abcam (Cambridge, MA); MG132 and purified 26S proteasome from BioMol (Plymouth Meeting, PA); fluorogenic proteasome substrates from Calbiochem (San Diego, CA); tetrahydro-L-biopterin dihydrochloride (BH4) from Cayman (Ann Arbor, MI). HUVECs and HMVEC were obtained from Cascade Biologics (Walkersville, MD) and ScienCell (Carlsbad, CA), respectively. Human GTPCH I antibody was kindly provided by Dr. Gabriele Werner-Felmayer (Innsbruck Medical University, Austria). All the other antibodies and reagents, including angiotensin II (Ang II) and streptozotocin (STZ), were obtained from Santa Cruz Biotechnology (Santa Cruz, CA) or Fisher Scientific (Pittsburgh, PA).

### Mice

Ten-week-old male C57BL/6J mice and low density lipoprotein receptor knockout (LDLr^−/−^) mice were obtained from the Jackson Laboratory (Bar Harbor, Me). Mice were housed in temperature controlled cages with a 12-hour light/dark cycle and given free access to water and chow. The mice were euthanized with inhaled isoflurane at the end of the animal experiments. Aortas were then removed for endothelial function assay or immediately frozen in liquid nitrogen for other assays. The animal protocols for models of diabetes, hypertension and dyslipidemia used in this paper were reviewed and approved by the Institutional Animal Care and Use Committee at the University of Oklahoma Health Sciences Center. The approved IACUC protocol numbers are: 10-153-H, 11-072-H and 11-045.

### Assays of the 26S proteasome activity

26S proteasome activity was assayed by measuring ATP dependent degradation of proteasome fluorescence substrate, as described previously [11], [14].

### Streptozotocin-induced diabetes mellitus in mice

A low-dose of STZ induction regimen was used to induce pancreatic islet cell destruction and persistent hyperglycemia as described by the Animal Models of Diabetic Complications Consortium (http://www.amdcc.org). Hyperglycemia was defined as a random blood glucose level of >450 mg/dL for >2 weeks after injection. One additional group of STZ mice received Tempol (Sigma; 1 mmol/L) in their drinking water for an additional 2 weeks. Aortas were all harvested 3 weeks after STZ injection.

### Ang II-induced hypertension and blood pressure measurement

Ang II was continuously administered in 10-week-old C57BL/6J mice (Jackson Laboratory, Bar Harbor, ME) at a rate of 0.8 mg/kg/d for 14 days using a mini-osmotic pump (Alzet®) as previously reported [15]. Arterial blood pressure was determined using a carotid catheter method as previously described [16]. High blood pressure (hypertension) was defined and achieved as previously reported [16]. Transfection with siRNA was performed as previously described [16].

RETRACTED

### LDLr^−/−^ dyslipidemia model

The LDLr^−/−^ mice were fed a Western diet or high fat diet (HFD) containing 0.21% cholesterol and 21% fat (Research Diets Inc, D12079B) for 8 weeks. Two weeks after HFD, an MG132 osmotic pump (delivered at rate of 0.72 mg/kg per day; DURECT Corporation, Model 2006) or the inhibitor-diluents (DMSO), as a negative control, was implanted subcutaneously in LDLr^−/−^ or the control WT mice for 6 weeks. Dyslipidemia was defined as previously reported [17].

### Assays of endothelium-dependent and endothelium-independent vasorelaxation

Vessel Aortic rings isolated from the treated mice were subjected to organ chamber assay of endothelium-dependent and -independent vasodilatation as described previously [11].

### Statistical analysis

Comparison of vasodilatation or data from other experiments involving more than two factors (such as endothelial dependent vessel relaxation assay) was performed with a two-way ANOVA, and intergroup differences were determined using the Bonferroni inequality method. All other results were analyzed with a one-way ANOVA. Values are expressed as mean ± SEM. P<0.05 was accepted as significant.

## Results

### Exogenous ONOO^−^ increase PA700 tyrosine nitration and 26S proteasome activity *in vitro*

To test the impacts of ONOO^−^ on the 26S proteasome, purified 26S proteasomes were exposed to low concentration (1 µM) of chemically synthesized ONOO^−^ *in vitro*. As depicted in Fig. 1, ONOO^−^ markedly increased 3-nitrotyrosine staining of PA700/S10B, the regulatory unit of 26S proteasome, without changing the apparent integrity of the proteasome (Fig. 1A). The increment of tyrosine nitration in PA700/S10B was correlated with an over 2-fold increase in 26S proteasome activity (Fig. 1B). Increased 26S proteasome activity was further confirmed by an *in situ* substrate-in-gel assay, in which the vehicle- or ONOO^−^ - treated 26S proteasomes were separated on a native-PAGE (3–14% gradient gel) followed by fluorogenic substrate incubation and fluorescence capturing under UV (Fig. 1C: in-gel substrate).

**Figure 1:** ONOO^−^ nitrates PA700/S10B and increases 26S proteasome activity both *in vitro* and in intact cell. *In vitro* (A–C): ONOO^−^ (1 µM) was incubated with the purified 26S proteasome for 5 min; in intact cell (D–E): HUVEC was incubated with ONOO^−^ for 0.5 h, in the presence or absence of uric acid (50 µM pre-incubation for 1 h). Cell free system (*in vitro*) was subjected to (A) Western blot to detect levels of PA700/S10B and the tyrosine nitration of 26S proteasome/PA700/S10B, (B) 26S proteasome activity (chymotrypsin-like activity), (C) an alternative 26S proteasome activity assay: a substrate-in-gel assay with a fluorogenic substrate followed by fluorescence capturing under the UV light. HUVEC cell lysate was subjected to (D) Western blotting of PA700/S10B tyrosine nitration and (E) assay of 26S proteasome activity (chymotrypsin-like activity). All blots shown are representative of three independent experiments. All results (n = 3) were analyzed with a one-way ANOVA.

RETRACTED

### ONOO^−^ nitrates PA700/S10B and increases 26S proteasome activity in intact endothelial cells

We next investigated if the effects of ONOO^−^ on proteasome activity could be recapitulated in HUVEC. As depicted in Figure 1D, exogenous addition of ONOO^−^ in HUVEC significantly enhanced tyrosine nitration of PA700/S10B compared to those treated with vehicle. Pre-incubation of uric acid (UA), a known ONOO^−^ scavenger, abolished the ONOO- enhanced PA700/S10B tyrosine nitration (Fig. 1D). Further, UA abrogated ONOO^−^ enhanced proteasome activation in HUVEC (Fig. 1E). In sum, these data suggest that exogenous ONOO^−^ causes tyrosine nitration of PA700/S10B resulting in consequent activation of 26S proteasome in HUVEC.

### ONOO^−^ enhances 26S proteasome assembly *in vitro* and in intact endothelial cells

The assembly of 19S and 20S proteasomes into 26S proteasome is considered as a key step in controlling 26S proteasome activity [5]. Thus, it was interesting to evaluate if ONOO^−^ increased the assembly of 19S and 26S proteasome sub-complexes. We first tested this on the purified proteasomes. We used native PAGE gel to separate the treated 26S proteasomes, like Fig. 1C, and then either performed a Western blotting (Fig. 2A: IB) or a direct staining with Coomassie Brilliant Blue (CBB) (Fig. 2A: CBB staining). Compared to the vehicle-treated (Fig. 2A), ONOO^−^-treated 26S proteasomes presented an increase in PA700/S10B IB staining as well as the 26S proteasome CBB staining, suggesting an increased 26S proteasome assembly (Fig. 2A: IB and CBB staining), which may contribute to the enhanced 26S proteasome activity (Fig. 1B and 1C).

**Figure 2:** ONOO^−^ promotes 26S proteasome assembly both *in vitro* and in intact cell. *In vitro* (A): ONOO^−^ (1 µM) was incubated with the purified 26S proteasome for 5 min; in intact cell (B): HUVEC was incubated with ONOO^−^ for 0.5 h, in the presence or absence of uric acid (50 µM pre-incubation for 1 h). Cell free system (*in vitro*) was subjected to (A) separation on a native gradient (3–14%) PAGE gel followed either by Western-blotting (IB) or a direct staining with coomassie brilliant blue (CBB staining) for 26S proteasome assembly. HUVEC cell lysate was subjected to (B) Western blotting of the PA700/S10B co-immunoprecipitates with a β7 antibody. All blots shown are representative of three independent experiments. All results (n = 3) were analyzed with a one-way ANOVA.

RETRACTED

We further tested if the ONOO^−^-mediated 26S proteasome assembly could be reproduced in intact cells. To avoid the confound effects exerted by the proteasome purification and enrichment which is required in the native gel approach, we adapted a previously described approach [12] by measuring the association of proteasome representative subunits to estimate 26S proteasome assembly. These subunits represent the19S (PA700/S10B) and the 20S (β7) sub-complex, respectively. As shown in Fig. 2B, ONOO^−^ increased 26S proteasome assembly, as evidenced by increased association of PA700/S10B and β7 subunits, compared to those treated with the vehicle. Pre-incubation of uric acid abrogated ONOO^−^-enhanced proteasome association in HUVEC (Fig. 2B). Collectively, these data suggest that exogenous ONOO^−^ promotes 26S proteasome assembly in intact cell.

### The 26S proteasome is activated in aortic homogenates from mouse models of diabetes, hypertension, and dyslipidemia

We sought to exploit if ONOO^−^-mediated 26S proteasome activation could be recapitulated in whole animals when cardiovascular risk factors were present. We first assayed 26S proteasome activity in mouse model of STZ-induced diabetes, Ang II-induced hypertension, and HFD induced dyslipidemia, which are all recognized cardiovascular risk factors and associated with oxidative stress. As shown in Fig. 3, homogenates from STZ-diabetic aorta presented a ∼2 fold increase in 26S proteasome activity compared to those of the vehicle-treated control mice (Fig. 3A). Injection of a potent proteasome inhibitor MG132 (5 mg/kg body weight, i.p. 2d., as reported [11], [18]) significantly decreased 26S proteasome activity in STZ-induced diabetic mice (Fig. 3A). In aortic preparation from Ang II-infused hypertensive mice, about 2-fold of increase in 26S proteasome activity were detected (Fig. 3B); however, knockdown of PA700/S10B, which were confirmed in Fig. 4B, suppressed the 26S proteasome activation (Fig. 3B). Similarly, compared to normal chow fed mice, aortic tissues prepared from HFD fed mice (dyslipidemia) presented approximately 2 fold increase in 26S proteasome activity (Fig. 3C); the enhanced 26S proteasome activation was blocked when MG132 was administrated (through the implanted osmotic pump with infusion rate of 0.72 mg/kg/d, 6 wks, as reported [19]) (Fig. 3C).

RETRACTED

**Figure 3:** The 26S proteasome is activated and results in degradation of the target proteins, which can be prevented either by ONOO^−^ inhibition or by MG132 administration, in aortic homogenates from mouse models of diabetes, hypertension, and dyslipidemia. Mouse models of (A) diabetes (STZ: 50 mg/kg/d, sham: sodium citrate, i.p., 5d; MG132, 5 mg/kg/d, i.p., 2d; n = 5/group); (B) hypertension (angiotensin II: 0.8 mg/kg/d, sham: saline; osmotic pump infusion, 14d.; PA700/S10B/control siRNA, i.v. 7d; n = 5/group) and (C) high fat-diets-induced atherosclerosis (LDLr^−/−^ mice, normal chow or HFD, 8 wks; MG132: 0.8 mg/kg/d; sham: saline; osmotic pump infusion, 2 wks after HFD, 6 wks; n = 5/group). AT the end of the animal experiment, aortas were removed and their homogenates were either subjected to 26S proteasome activity assay (chymotrypsin-like activity) (A–C), or Western blotting with the corresponding antibodies as indicated. All results (n = 5) were analyzed with a one-way ANOVA. * indicates significant *vs.* control; NS: not significant *vs*. control.

**Figure 4:** PA700/S10B tyrosine nitration and 26S proteasome sub-complex association (assembly), but not the PA700/S10B protein levels, are increased in aortic homogenates from mouse models of diabetes, hypertension, and dyslipidemia. Mouse models of (A) diabetes (STZ: 50 mg/kg/d, sham: sodium citrate, i.p., 5d; Tempol, 1 mmol/kg/drinking water, 2 wks.; n = 5/group); (B) hypertension (angiotensin II: 0.8 mg/kg/d, sham: saline; osmotic pump infusion, 14d.; PA700/S10B/control siRNA, i.v. 7d; n = 5/group) and (C) high fat-diets-induced dyslipidemia (LDLr^−/−^ mice, normal chow or HFD, 8 wks; MG132: 0.8 mg/kg/d; sham: saline; osmotic pump infusion, 2 wks after HFD and for 6 wks; n = 5/group). AT the end of the animal experiment, aortas were removed and their homogenates were subjected to immunoprecipitation and Western blot. The immunoprecipitation assay was performed using either an anti-PA700/S10B or anti-3-NT antibody. All blots shown are representative for mice n = 5. All results were analyzed with a one-way ANOVA. * indicates significant *vs.* control; NS: not significant *vs*. control.

### Pharmacologic or genetic inhibition of 26S proteasome prevents GTPCH I and thioredoxin from degradation in mouse models of diabetes, hypertension, and dyslipidemia

We next exploited the functional outcomes of the altered 26S proteasome activity by examining the turnover of proteins that are essential to endothelial cell homeostasis and are recognized substrates of or related to the 26S proteasome. GTP cyclohydrolase I (GTPCH I) is one of the very few known proteins in this category. As a potential substrate of the 26S proteasome [11], [20], [21], [22]_ENREF_23, GTPCH I is a rate limiting enzyme for *de novo* synthesis of tetrahydrobioptin (BH4), a key cofactor of eNOS [23]. Indeed, aortas from diabetic (Fig. 3D), hypertensive (Fig. 3E) mice, but not the control mice, presented decreased GTPCH I levels, as we previously reported [11], [12]. Interestingly, protein levels of GTPCH I were also found decreased in aortic tissues from the HFD-induced dyslipidemia mice, compared to normal chow fed mice (Fig. 3F). Furthermore, protein levels of thioredoxin (Trx), a protein important to maintain a cellular reducing environment [24], [25], was also decreased in aortas from the mice of diabetes (Fig. 3D), hypertension (Fig. 3E), and dyslipidemia (Fig. 3F). Importantly, inhibition of ONOO^−^ generation by Tempol administration (Fig. 3D), or inhibition of the 26S proteasome by siRNA-mediated PA700/S10B knockdown (Fig. 3E), or by MG132 treatment, restored protein levels of both GTPCH I and Trx (Fig. 3D, 3E, and 3F).

RETRACTED

### Enhanced PA700/S10B tyrosine nitration and 26S proteasome assembly in mouse models of diabetes, hypertension, and dyslipidemia

We then investigate the potential mechanisms underlying 26S proteasome activation which would be shared by all studied models. To this end, we used an anti-PA700/S10B antibody to pull down PA700/S10B so that the levels of nitrated PA700/S10B could be assessed with an anti-nitrotyrosine antibody in Western blot. As shown in Fig. 4A, compared to those of vehicle-treated mice, aorta from the STZ-treated mice presented higher levels of PA700/S10B tyrosine nitration, accompanied by enhanced 26S assembly, as evidenced by increased association of 26S proteasome sub-complexes (PA700/S10B, the 19S proteasome sub-complex and the 20S proteasome core), but not PA700/S10B protein levels (Fig. 4A). Importantly, these augments were abolished in mice treated with Tempol, a potent superoxide scavenger therefore an inhibitor of ONOO^−^ generation (Fig. 4A).

Like the effect of STZ-induced diabetes, Ang II also increased PA700/S10B tyrosine nitration and 26S proteasome assembly, but not PA700/S10B protein levels (Fig. 4B), consistent with our previous studies [12]. Furthermore, siRNA-mediated PA700/S10B knockdown prevented association of 26S proteasome sub-complexes as expected (Fig. 4B). Such a loss of 26S proteasome assembly was in line with the blockage of Ang II-induced 26S proteasome activation (Fig. 2B) and of the reduction of GTPCH I and Trx protein levels (Fig. 3B).

Importantly, HFD, but not the normal chow feeding, elevated both PA700/S10B tyrosine nitration and 26S proteasome assembly (Fig. 4C). Interestingly, MG132 infusion for 6 weeks reversed these increase, without affecting PA700/S10B protein levels (Fig. 4C). Of note, the levels of PA700/S10B tyrosine nitration and 26S proteasome assembly were closely related to those of the 26S proteasome activity (Fig. 3C).

RETRACTED

### Nitration of PA700/S10B-mediated 26S proteasome induces endothelial dysfunction

Finally, we monitored the endothelial function of isolated vessel, a valuable surrogate endpoint to assess the impact of therapeutic interventions [26]. As presented in Fig. 5, aortas from diabetic but not control mice, exhibited impaired acetylcholine-induced vessel relaxation (Fig. 5A) in parallel with a down-regulation of both GTPCH I and Trx proteins (Fig. 3D), which were associated with enhanced PA700/S10B tyrosine nitration, 26S proteasome assembly (Fig. 4A) and activation (Fig. 3A). However, these effects were abolished when Tempol, a SOD mimetic, was co-administrated (Fig. 3D, 4A, and 5A), a reminiscence of the protective effect of MG132 administration previously observed [11]. In contrast, aortas from all group of mice presented no significant differences in vessel relaxation evoked by sodium nitroprusside (SNP) (Fig. 5B), an NO donor that can induce endothelium-independent vessel relaxation [27]. This indicates that the impairment of acetylcholine-induced vessel relaxation is mainly due to endothelial dysfunction.

**Figure 5:** Inhibition of the 26S proteasome either by ONOO^−^ inhibition or by MG132 administration rescues endothelial dysfunction in mouse models of diabetes, hypertension, and dyslipidemia. Mouse models of (A/B) diabetes (STZ: 50 mg/kg/d, sham: sodium citrate, i.p., 5d; Tempol, 1 mmol/kg/drinking water, 2 wks.; n = 5/group); (C/E) hypertension (angiotensin II: 0.8 mg/kg/d, sham: saline; osmotic pump infusion, 14d.; PA700/S10B/control siRNA, i.v. 7d; n = 5/group) and (D/F) high fat-diets-induced dyslipidemia (LDLr^−/−^ mice, normal chow or HFD, 8 wks; MG132: 0.8 mg/kg/d; sham: saline; osmotic pump infusion, 2 wks after HFD and for 6 wks; n = 5/group). AT the end of the animal experiment, aortas were removed for endothelial function assay. The removed aortas were cut into 3-mm rings, and precontracted with 30 nmol/L of U46619 in organ chambers (PowerLab, ADInstruments, Colorado Springs, Co). (A/C/D) Endothelium-dependent vasodilator responses were determined in the presence of acetylcholine (0.01 to 100 µmol/L). (B/E/F) Endothelium-independent vasodilator responses were determined in the presence of sodium nitroprusside (SNP) (0.0001 to 1 µmol/L). All results were analyzed with a one-way ANOVA. * indicates significant *v.s.* control; NS: not significant *v.s.* control.

Similarly, aortas from the mice of Ang II-induced hypertension (Fig. 5C) and of HFD-induced dyslipidemia (Fig. 5D) shared the same pathway, manifesting as an impaired acetylcholine-induced vessel relaxation (Fig. 5C and 5D) which were associated the PA700/S10B-mediated 26S proteasome activation (Fig. 3B, 3C, 4B, and 4C). Most importantly, inhibition of the 26S proteasome either by siRNA-mediated PA700/S10B knockdown (Fig. 5C) or by MG132 administration (Fig. 5D) significantly ameliorated the acetylcholine-induced vessel relaxation. Likewise, there were no significant differences in SNP-evoked vessel relaxation among groups (Fig. 5E and 5F), further indicating that endothelial dysfunction contributes to the impaired vessel relaxation.

RETRACTED

## Discussion

In this study, we have defined a mechanism shared by different models of cardiovascular diseases, in which tyrosine nitration of PA700/S10B- mediated 26S proteasome deregulation is linked to endothelial dysfunction, a key surrogate marker for CVD. To the best of our knowledge, this is the first report on the impacts of oxidative stress on a major subcellular system in multiple animal models with risk factors of cardiovascular disease. Proteasome deregulation could alter essential cellular targets, resulting in diseased conditions (Fig. 6). Therefore, the current study will open new avenue to proteasome-related mechanisms in CVD.

**Figure 6:** Tyrosine nitration of PA700/S10B-mediated proteasome activation is a common pathway leading to endothelial dysfunction in mouse models with cardiovascular risk factors. Oxidative stress plays an essential role in the parthenogenesis of cardiovascular diseases including diabetes, hypertension and dyslipidemia. ONOO^−^, formed by the reaction of superoxide with nitric oxide at diffusion-controlled rate, when overproduced, has been demonstrated to affect various pathophysiological events. The presented evidence support a shared mechanism in mouse models with cardiovascular risk factors, in which deregulation of 26S proteasome caused by ONOO^−^, likely via tyrosine nitration of PA700/S10B, the regulatory complex of 26S proteasomes. Proteasome deregulation could alter essential cellular targets, resulting in early diseased conditions, such as endothelial dysfunction (the initial damaging stage), which may either adaptively improve or worsen the conditions (arrows). Identification of mechanisms underlying these alterations may help to define proper intervention to bring clinic benefit to the patients.

In supporting the notion that oxidative stress links 26S proteasome activation to endothelial dysfunction, we have provided evidence at various setting ranging from cell free and cell culture to whole animal models with common CVD risk factors. In highlights, we found that (1) ONOO^−^ reacts directly with the isolated 26S proteasome, which results in increased 26S proteasome assembly and activation, likely through the enhanced tyrosine nitration of PA700/S10B, the key regulatory complex of 26S proteasomes; (2) such a ONOO^−^-mediated biochemical process occurs in intact culture cells, because pretreatment of the culture cells with UA, a ONOO^−^ scavenger, prevents the 26S proteasome activation pathway; (3) independent of the type of CVD risk factors in the studied models, aortic 26S proteasome activation are all present; (4) the 26S proteasome activation in animal study manifests as the increased 26S proteasome assembly and activity, which are all accompanied by augmented PA700/S10B tyrosine nitration; (5) activation of aortic 26S proteasome decreases proteins which are important to endothelial homeostasis; such as GTPCH I, which is directly related to NO bioavailability and key to the vascular endothelial function, and Trx, which is related to endothelial function maintenance [24] through reactive oxygen species scavenging [28], apoptosis suppression [29], or survival promotion [30]; (6) intervention through ONOO^−^ inhibition (Tempol administration) or through 26S proteasome inhibition, via pharmaceutical (MG132 administration) or genetic approaches (siRNA knockdown of PA700/S10B), restore GTPCH I and Trx, the proteins that have been shown important for endothelial homeostasis; (7) these data are further validated in vivo in that either inhibition of endogenous ONOO^−^ or 26S proteasome activation could ameliorate the otherwise impaired endothelial function (restoration of acetylcholine-induced vessel relaxation). Emerging data support that proteasome assembly, including 26S complex assembly [6], [31], [32] and individual sub-complex assembly [33], [34], is important for its function. Post-translational modifications of PA700 have been linked to the regulation of proteasome assembly [35] and function [36], although it remains to be established how tyrosine nitration observed in present study would affect the assembly. Therefore, the increased 26S assembly, induced by oxidative stress (e.g. ONOO^−^) mediated proteasome modifications (e.g. tyrosine nitration), is likely the mechanism for deregulated 26S proteasome, which is linked to endothelial dysfunction shared by the studied mouse models.

RETRACTED

A cardinal feature of endothelial dysfunction is impaired endothelium-dependent vasodilatation caused by loss of NO bioavailability [37]. Not a single mechanism alone can explain endothelial dysfunction. Rather, an interplay among multiple regulatory pathways results in pathogenesis of this vascular disorder [38], [39], [40]. Oxidant such as ONOO^−^ attacks various molecules in vascular endothelium, vascular smooth muscle and myocardium, eventually leading to endothelial dysfunction in CVD [2]. In the present study, GTPCH I degradation is attributed to ONOO^−^ activated 26S proteasome in several models. However, we did not exclude the possibility that ONOO^−^ also makes it a good substrate for proteasome, since mild modification by ONOO^−^ results in selective recognition and degradation by proteasome [41]. In either case, activated 26S proteasome would accelerate GTPCH I degradation. It is crucial to maintain appropriate levels of GTPCH I protein for vascular health, since GTPCH I deficiency has been demonstrated in animal models to cause endothelial dysfunction [11] and high blood pressure [16]. In contrast, restoration of GTPCH I has been found beneficial [42], which is due, at least in part, to the improved endothelial function [42], [43] or the suppression of oxidative stress [44]. It is intriguing that the proteins responsible for redox regulation, such as Trx, are in the list of the proteasome substrates in the present study. These proteins have been shown to be endothelial function protective. For instance, the predominant role of Trx to limit oxidative stress directly has been demonstrated in various disease models [45]. Although we presented limited target proteins as evidence of functional proteasome activation, we expect other key molecules may undergo the same pathway which warrants further investigation. In fact, increasing evidence revels that UPS involves in the turn-over of eNOS [46], [47], [48], [49], one of the most endothelial protective molecule, and several other factors essential to endothelium homeostasis [50]. It is widely believed that imbalance between the generation of endothelial-derived relaxing factors (EDFR) and contracting factors (EDCF) may contribute to endothelial dysfunction [51]. Therefore, it would be important to examine if UPS also affects the turnover of these factors globally, an under-examined dimension of proteomics in protein stability in humans [52]. It is also important to note that global activation of 26S proteasome does not guarantee target degradation, a complex process that may require additional (co)factors. However, given the fact that PA700/S10B siRNA knockdown abolishes the effects mediated by proteasomes, 26S proteasome activation does play a decisive role in the degradation of its substrates. In any case, the observed activation of 26S proteasome may be one of the crucial partners for the whole degradation process. It merits further investigation to identify new partners in this unified mechanism.

RETRACTED

In summary, the preclinical data presented here indicate that oxidative stress (ONOO^−^) might be the common linker that connects 26S proteasome activation to endothelial dysfunction, which is prevalent in most types of CVD. Although targets of ONOO^−^ vary [2]_ENREF_2, manipulating the shared one as demonstrated in this study may bring overall beneficial clinic outcome. The findings in this study also may provide insight to drug design for CVD in that targeting specific components of the 26S proteasome might improve the outcomes of medical intervention.
